# Potential Mechanisms of White Peony against Primary Sjögren's Syndrome Based on Network Pharmacology and Molecular Docking

**DOI:** 10.1155/2022/5507472

**Published:** 2022-08-12

**Authors:** Shuqi Zhuang, Jincheng Pu, Yuanyuan Liang, Zhenzhen Wu, Ronglin Gao, Shengnan Pan, Jiamin Song, Jianping Tang, Xuan Wang

**Affiliations:** Department of Rheumatology and Immunology, Tongji Hospital, School of Medicine, Tongji University, Shanghai 20065, China

## Abstract

**Background:**

Multiple system and organ damage occurs with the continuous progression of primary Sjögren's syndrome (pSS), and the lack of specific drugs against this disease is a huge challenge. White peony (WP), a widely used traditional Chinese herb, has been confirmed to have a therapeutic value in pSS. However, the specific mechanisms of WP in the treatment of pSS are unknown.

**Methods:**

The active ingredients and their targets in WP were searched on the Traditional Chinese Medicine Systems Pharmacology Database and Analysis Platform (TCMSP), and disease-related targets were collected from GeneCards, Online Mendelian Inheritance in Man (OMIM), and the Therapeutic Target Database (TTD). The overlapping targets were acquired by taking the intersection. A protein-protein interaction (PPI) network was structured using the STRING database. A disease-drug-ingredient-target (D-D-I-T) network was built using Cytoscape software. By filtering twice, core targets were acquired. Gene Ontology (GO) and Kyoto Encyclopedia Gene and Genome (KEGG) pathway enrichment analysis were accompanied by R packages. Finally, molecular docking was used to verify the abovementioned results.

**Results:**

In total, we screened 88 WP-related targets, 1480 pSS-related targets, and 32 overlapping targets. D-D-I-T Network analysis displayed six main active ingredients of WP, which played a significant therapeutic role in pSS. Further topological analysis selected seven core target genes, including IL-6, TNF, PPAR*γ*, AKT1, CASP3, NOS3, and JUN. GO and KEGG analysis were used to elucidate pharmacological mechanisms, mainly acting in the AGE-RAGE signaling pathway. Molecular docking proved that paeoniflorin bound well with core targets.

**Conclusion:**

Our study revealed that IL-6, TNF, AKT1, CASP3, NOS3, and JUN may be pathogenic target genes, and PPAR*γ* may be a protective target gene. The main active ingredients of WP mainly played a therapeutic role via the AGE-RAGE signaling pathway. These findings provide a fundamental and theoretical basis for the clinical application of WP.

## 1. Introduction

Primary Sjögren's syndrome (pSS) is a systemic autoimmune disease, and the majority of patients are female, aged approximately 50 years. The global incidence of pSS is 6.92 per 100,000 person-years, with a prevalence of 60.82 cases per 100,000 people [1]. Objective oral and ocular mucosal dryness are the hallmarks of pSS and are due to lymphocytic infiltration of exocrine glands, primarily salivary, and lachrymal glands, which leads to secretory dysfunction. In addition, fatigue, limb pain, and other nonspecific symptoms can also occur during the disease course [2]. In the advanced stage, systemic complications can develop, including B-cell lymphoma, interstitial lung disease, and peripheral neuropathy, which can result in reduced working ability, poor quality of life, increased mortality, and greater financial burden on the patient's family. The pathological mechanism of pSS is complex and not fully explained; however, it is agreed that both innate and adaptive immune responses are involved in the occurrence and development of the disease [3]. To date, due to the lack of specific and effective drugs, immunomodulatory drugs including prednisone, hydroxychloroquine, methotrexate, mycophenolate sodium, azathioprine, and cyclosporine are administered as conventional medicines in clinical practice for the treatment of pSS, based on the guidelines for systemic lupus erythematosus (SLE) and other connective tissue diseases [4]. However, the beneficial effects of these medicines are limited and patients can experience obvious side effects [5]. Biologic agents recently used for targeted therapy have expanded our treatment strategy. Although several biologic agents are available for pSS treatment, none have provided satisfactory efficacy [6]. Treatment with traditional Chinese medicine has a time-honored history, with a multicomponent, multipathway, multitarget therapeutic mode. It is readily available, inexpensive, safe, and effective. The comprehensive application of traditional Chinese medicine is worth further investigation.

Radix Paeoniae Alba (RPA), is also called white peony (WP) in China. As a traditional Chinese medicine, it is derived from the radix of Paeonia of *Ranunculaceae*. Total glucosides of peony (TGP), extracted from RPA, consist of paeoniflorin (Pae), albiflorin, hydroxyl-paeoniflorin, benzoylpaeoniflorin, benzoyloxypeoniflorin, and others [7]. Pae is a crucial component of TGP and possesses extensive anti-inflammatory, antioxidative, and immune regulatory effects [7, 8]. TGP capsule, branded as Pavli, was approved by China Food and Drug Administration (CFDA) to treat rheumatoid arthritis (RA) in 1998 [9]. In addition, it is also used to treat SS, psoriasis, and other immune-dysregulated diseases in modern clinical practice. A largescale Chinese survey showed that the utilization rate of TGP in SS patients was 41.7% [10]. Other research studies demonstrated that TGP monotherapy in pSS was effective [11, 12], and co-administration of TGP with an immunosuppressant (IS) showed superior therapeutic efficacy than IS alone [13], which mainly manifested in ameliorating sicca symptoms, reducing the local concentration of autoantigens, and decreasing the serum level of inflammatory cytokines [11, 12, 14]. Furthermore, the most common adverse effects (AEs) of TGP were diarrhea and gastrointestinal discomfort [13], which were less severe compared with other conventional medicines for pSS. However, its clinical application is hampered due to its complex chemical composition and lack of data on its underlying mechanisms.

Network pharmacology is a novel paradigm in drug discovery based on the rapid progress of interdisciplinary fields such as bioinformatics and systems biology [15]. Molecular docking can predict the interactions between ligands and receptors at the molecular level [16]. In the present research, network pharmacology was adopted to identify the active ingredients of WP, screen potential therapeutic targets, and explore potential signaling pathways of WP against SS. In addition, molecular docking was employed to analyze the optimal active ingredients (Figure 1). Consequently, this research illustrates the underlying mechanism of WP in the treatment of pSS and provides a broad platform for research into new drugs.

## 2. Materials and Methods

### 2.1. Potential Therapeutic Targets

In order to verify that the intrinsic ingredients in TGP are valuable and to identify other new compounds, we searched the ingredients of WP on the Traditional Chinese Medicine Systems Pharmacology (TCMSP) database (https://tcmspw.com/tcmsp.php). To obtain the main active ingredients with superior pharmacological properties based on ADME (absorption, distribution, metabolism and excretion), two parameters were required: (1) oral bioavailability (OB) ≥ 30% and (2) drug-likeness (DL) ≥ 0.18 [17]. In addition, related target genes were extracted. Subsequently, these target gene names were calibrated to avoid deviation using the UniProt database (https://www.uniprot.org/) under the condition of “*Homo sapiens”*. Disease-related target genes were downloaded and merged from the GeneCards database (https://www.genecards.org/), Online Mendelian Inheritance in Man (OMIM) (https://omim.org/search/advanced/geneMap) and the Therapeutic Target Database (TTD) using the keyword “Sjögren's Syndrome” [17, 18]. The revised and overlapping target genes, which were viewed as potential therapeutic target genes, were acquired by taking an intersection between the drug-related and the disease-related using the Venny tool (https://bioinfogp.cnb.csic.es/tools/venny/index.html).

### 2.2. Protein-Protein Interactions (PPI) Network and Disease-Drug-Ingredient-Target (D-D-I-T) Network Construction

The overlapping target genes were transferred into the STRING database (https://cnstring-db.org/cgi/input.pl) to predict interactions between the genes by setting the organism to “*Homo sapiens*”. Therefore, a PPI network graphic could be constructed, where nodes represented genes and edges represented gene-gene associations [19]. Then, a D-D-I-T network map was established and visualized via Cytoscape software (version 3.9.0) to display the relationships between components and targets. A “CytoNCA” plugin was used to select the core targets, after two cycles of screening where the betweenness centrality (BC), closeness centrality (CC), and degree centrality (DC) were limited to greater than the medians [20].

### 2.3. Gene Ontology (GO) Biological Functions and Kyoto Encyclopedia Gene and Genomes (KEGG) Pathway Enrichment Analysis

In the R working environment, the core target gene symbols were translated into Entrez ID. Then, to predict potential pharmacological mechanisms of WP against SS, GO and KEGG pathway enrichment analyses were performed, respectively [21]. A *P* value <0.05 was considered statistically significant.

### 2.4. Molecular Docking

The 2D structures of the main active ingredients were downloaded from the PubChem database (https://pubchem.ncbi.nlm.nih.gov/) and converted into 3D structures using Chem3D software (version 20.0). Through energy minimization calculations, these structures were saved in the mol2 format [22]. The 3D structures of core target genes were obtained from the RCSB PDB database (https://www.rcsb.org/). The AutoDockTools software (version 1.5.7) completed file format conversion to pdbqt format, and active pocket coordinates determination. The affinities between ligands and receptors were evaluated as docking energies by AutoDock Vina software (version 1.2.0). They were considered to bind well with each other when the docking energy was less than −5 kcal/mol [23]. The PyMOL software (version 2.5.2) implemented molecular docking and nonpolar hydrogen addition exhibition.

## 3. Results

### 3.1. Potential Therapeutic Targets

According to the “Baishao” search in the TCMSP database, we identified 85 ingredients. Screened by OB ≥ 30% and DL ≥ 0.18, 13 active ingredients were ultimately established (5 of them lacked related target genes). They were 11alpha,12alpha-epoxy-3beta-23-dihydroxy-30-norolean-20-en-28,12beta-olide, paeoniflorgenone, (3S, 5R, 8R, 9R, 10S, 14S)-3, 17-dihydroxy-4, 4, 8, 10, 14-pentamethyl-2, 3, 5, 6, 7, 9-hexahydro-1H-cyclopenta(a)phenanthrene-15, 16-dione (DPHCD), lactiflorin, paeoniflorin, paeoniflorin_qt, albiflorin_qt, benzoyl paeoniflorin, mairin, beta-sitosterol, sitosterol, kaempferol, and (+)-catechin (Table 1). Through calibration and screening for repeats in the UniProt database, a total of 88 drug-related target genes were ultimately obtained. A total of 1480 disease-related target genes were identified after merging and excluding duplicates from GeneCards, OMIM, and TTD. Finally, using the Venny tool, 32 overlapping targets, viewed as potential therapeutic targets were obtained and are shown in Figure 2(a).

### 3.2. Protein-Protein Interaction Network (PPI) and Disease-Drug-Ingredient-Target (D-D-I-T) Network Construction

The 32 overlapping target genes were imported into the STRING database and a PPI Network graphic was demonstrated (Figure 2(b)). There were 32 nodes and 185 edges in the graphic. The average node degree was 11.6, and the local clustering coefficient was 0.745. A D-D-I-T network map was constructed using Cytoscape software (Figure 3), where every active component acted on multiple targets and key targets also interacted with multiple active components. Further topological analysis filtered seven target genes, which were viewed as potential core targets with therapeutic effects on pSS (Figure 4). The top seven core targets, namely, interleukin-6 (IL-6), tumor necrosis factor (TNF), peroxisome proliferator-activated receptor gamma (PPAR*γ*), RAC-alpha serine/threonine-protein kinase (AKT1), caspase-3 (CASP3), nitric-oxide synthase, endothelial (NOS3), and transcription factor AP-1 (JUN) are listed in Table 2.

### 3.3. Gene Ontology (GO) Biological Functions and Kyoto Encyclopedia Gene and Genome (KEGG) Pathway Enrichment Analysis

The biological functions and potential therapeutic mechanisms of the target genes were acquired via GO and KEGG enrichment analysis (*P* value < 0.05). The top 20 GO items and top 20 KEGG pathways are shown in Figure 5(a) and 5(b)), which were ranked by the GeneRatio. When the bubble color is purple and the bubble size is larger, the enrichment degree is higher.

GO analysis results covered three biological levels-biological process (BP), cellular component (CC), and molecular function (MF). In total, 1089 items in BP, the targets mainly enriched in response to lipopolysaccharide, response to molecules of bacterial origin, regulation of smooth muscle cell proliferation, and others. Five items in CC mainly included membrane raft and membrane microdomain. Sixty items in MF mainly included cytokine receptor binding, R-SMAD binding, TNF receptor superfamily binding, and others. A total of 96 pathways were found, and many were closely related to pSS, such as the Advanced Glycation End Product-Receptor for AGE (AGE-RAGE) signaling pathway, TNF signaling pathway, IL-17 signaling pathway, apoptosis, etc. Furthermore, the associated target genes of the AGE-RAGE signaling pathway are presented in detail in Figure 6.

### 3.4. Molecular Docking

The top three key compounds (kaempferol, beta-sitosterol, and Pae) were selected to dock to seven core target genes in turn and their docking energies were calculated (Table 3). Lower docking energy indicated a stable interaction and a close affinity between ligand and receptor. Our results further proved the critical status of the aforementioned core targets in treating pSS with WP. Pae has been discovered to have therapeutic value in SS in many studies, and it was taken as an example to perform the docking experiments. As shown in Figure 7, there is a stable hydrogen bond between Pae and core target genes. Their docking energies also exhibited good affinities.

## 4. Discussion

Yin deficiency, dryness, and heat in the body are viewed as pathological mechanisms of pSS, while body fluid deficiency, qi-stagnation, blood stasis, and phlegmatic hygrosis are viewed as manifestations of pSS in traditional Chinese medicine [24]. WP is thought to have the functions of nourishing blood, arresting yin, and repressing liver yang [25] and is widely used in China. In western medicine, WP was found to have anti-inflammatory and immunoregulatory effects. Taking its complex chemical composition into consideration, the mechanism of WP is unclear.

We attempted to preliminarily investigate the possible pharmacological mechanisms of WP in treating pSS using network pharmacology and molecular docking. As shown by KEGG pathway analysis, the therapeutic targets are mainly enriched in AGE-RAGE, TNF, IL-17, Toll-like receptor, the c-type lectin-like receptor signaling pathway, and apoptosis, of which the most important is the AGE-RAGE signaling pathway. Advanced glycation end (AGE) products are the final products of nonenzymatic glycation and protein oxidation, and the level of these products has been found to increase in many autoimmune diseases, including SLE, severe psoriasis, and RA. In the AGE-RAGE signaling pathway, AGE, by binding with the multiligand receptor RAGE, transduces signals via several pathways: JAK2-STAT1, PI3K-AKT, MAPK-ERK, and NADPH oxidase-ROS, consequently resulting in NF-*κ*B activation, and leads to the generation of proinflammatory cytokines, the presence of oxidative stress and the maintenance of a sustained inflammatory state [26, 27]. A preliminary study found that RAGE was overexpressed in the salivary glands of SS patients, but its potential mechanism was not investigated [28]. Aota et al. carried out an in vitro experiment to prove that inhibition of the JAK2/STAT1 pathway can decrease the secretion of CXCL10 in human salivary gland ductal cells [29]. Similarly, the activation of the PI3K/Akt signal pathway was found in non-obese diabetic (NOD) mice, and the expression of phosphorylated PI3K and AKT protein was suppressed when treated with QZF (Qing Zao Fang, a traditional Chinese medicine) [30]. In addition, the RAGE expression can be induced by the activation of NF-*κ*B, resulting in a vicious cycle of dysregulated inflammatory responses.

Based on the D-D-I-P network, we eventually found that six key active ingredients, including Pae, (+)-catechin, kaempferol, sitosterol, beta-sitosterol, and DPHCD had therapeutic efficacy against pSS. The main ingredients interacting with core targets were Pae, kaempferol, and beta-sitosterol. Pae, considered a principal component of TGP, has been extensively studied. There is no uniform preparation process for TGP capsules in pharmaceutical companies, which leads to the production of specific compounds which are different; however, Pae accounts for at least 40% of TGP [8]. It influences autoimmunity and inflammation from multiple aspects, for example, it suppresses the proliferation of peripheral blood mononuclear cells (PBMCs), modulates the ratio of T helper type 17/regulatory T (Th17/Treg) cells, and depresses T and B lymphocytes activation [31–35]. These cells are generally accepted to participate in the pathological process of pSS. With regard to intracellular pathways, Pae regulates the MAPKs-NF-*κ*B, PI3K-Akt-TOR, and JAK2-STAT3 signaling pathways [8, 31]. The underlying mechanisms maintain high conformity with the downstream effects of the AGE-RAGE signaling pathway. Zhang et al. established a RAW264.7 cell model stimulated by AGEs, and treatment with Pae inhibited the overexpression of AGEs-induced proinflammatory cytokines in a dose-dependent manner [36]. Thus, Pae may act on the AGE-RAGE pathway. Moreover, another in vitro experiment found that Pae increased intracellular Ca^2+^ concentration through endogenous release in salivary gland cells, which may promote salivation [37]. The study by Kapil Suchal demonstrated that kaempferol had antioxidant activity by blocking the AGE-RAGE/MAPK axis in a diabetic rat model with myocardial ischemia-reperfusion. In this study, the NF-*κ*B pathway was inhibited, leading to a decrease in the release of inflammatory cytokines [38]. In a rat model of alcoholic liver injury, researchers found that beta-sitosterol could protect hepatic cells from oxidative stress and downregulate endogenous cell apoptosis via the PI3K/Akt pathway [39]. Furthermore, beta-sitosterol could also exert anti-inflammatory actions by repressing p38, ERK, and NF-*κ*B pathways, which has been verified by in vitro experiments [40]. Of the other three active ingredients that are not closely linked to core targets, both (+)-catechin and sitosterol have anti-inflammatory bioactivity. However, there is little research on DPHCD, and attention should be focused on this ingredient in the future, which may have potential in new drug development.

According to the series of filters for overlapping targets, IL-6, TNF, PPAR*γ*, AKT1, CASP3, NOS3, and JUN were viewed as core targets. IL-6 takes part in the progression of inflammation and immunity. Previously named cell stimulatory factor 2 (BSF-2), IL-6 performs an important function by inducing B-cell differentiation into plasma cells, leading to autoantibody production and hypergammaglobulinemia. In addition, IL-6 promotes the differentiation of naïve CD^4+^ T cells, linking the innate immune response to the acquired immune response [41]. Moreno-Quispe et al. found that the level of IL-6 was higher in saliva, and a salivary gland biopsy in pSS patients showed a positive correlation with the severity of xerostomia [42]. Other scientific research showed that an increase in circulating IL-6 levels was detected in SS patients, which was associated with systemic inflammatory indicators (ESSDAI, ESR, CRP, and IgG) [43]. Furthermore, the high level of IL-6 is related closely to interstitial lung disease (ILD), a complication of SS [44]. The inappropriate activation of TNF-*α* signaling can contribute to autoimmune diseases. The serum level of TNF-*α* is elevated in SS patients [45]. Other studies have shown that an TNF-*α* blocker had an antiapoptotic effect on human salivary gland epithelial cells which is a significant pathological environment for SS [46], and suppressed inflammation in the lacrimal gland and cornea in dry eye treatment [47]. Akt, functioning as protein kinase B, is a central protein in many cellular pathways such as the cell cycle, growth, survival, metabolism, and immunity. As an isoform, Akt1 has been proved to correlate with autoimmune diseases such as SLE and multiple sclerosis [48, 49]. The Akt1/mTOR signaling pathway is crucial for the IL-17 expression [50], which is involved in the pathogenesis of pSS. The IL-17 signaling pathway can upregulate the expression of inflammatory genes to amplify inflammation by activating the NF-*κ*B and MAPK pathway [51]. As a cytokine principally sourced from Th17 cells, it was reported to show abnormal expression and correlate with disease severity in SS [52]. In experimental NOD mice, IL-17 may affect salivary secretion by destroying salivary tight junction integrity [53]. CASP3 occupies a central position in programmed apoptosis due to proteolytic cleavage of a variety of key proteins. The activation of CASP3 has been detected in the SS mouse model [54]. NOS3 (also named eNOS) is expressed in conjunctival epithelium and is associated with the severity of dry eye symptoms in SS [55]. With regard to JunB, a member of the JUN family, it can regulate Th17 and Treg cells [56, 57]. Different to the abovementioned targets, PPAR*γ* has anti-inflammatory effects by degrading intrinsic NF-*κ*B. Other aspects of PPAR*γ* in immunity are that PPAR*γ* can inhibit the expression of Th1 and Th2 cytokines to control the progression of SS in NOD mice and suppress the proliferation and differentiation of Th17 cells, which mainly release IL-17 [58]. Existing studies have revealed that downregulation of PPAR*γ* was strongly relevant to lacrimal gland dysfunction in dry eyes [59].

Experimental evidence suggests that Pae can suppress the release of inflammatory cytokines, such as IL-6 and TNF-*α* [60]. Furthermore, in rats with collagen-induced arthritis, Pae was proved to reduce phosphorylated Akt, resulting in decreased production of antibodies [35]. Lu et al. [61] revealed that Pae had a protective function by upregulating PPAR*γ* and displayed an antiapoptotic effect by downregulating CASP3 and Bax. Kaempferol treatment reduced the expression of NOS3 and TNF-*α*, which mainly modulated the NF-*κ*B and MAPK pathways in a rat model [62]. Beta-sitosterol can act on these targets leading to similar effects.

As a result, molecular docking reflected a strong affinity between three key ingredients of WP and seven core target genes. Our results describe the synergistic effects between ingredients and targets and emphasize the multicomponent, multipathway, and multitarget therapeutic mode of traditional Chinese medicine. However, our research also has certain limitations. What we predicted in theory, with the exception of DPHCD, can be supported more or less by existing research, but it is hoped that more in vivo or in vitro experiments can further strengthen our conclusions. In terms of DPHCD, which has been rarely studied, this compound may provide potential for the development of new drugs.

## 5. Conclusion

In summary, WP has a significant advantage in the treatment of pSS, which is consistent with previous studies. Kaempferol, beta-sitosterol, and paeoniflorin in WP have therapeutic effects against pSS by inhibiting six targets, including IL-6, TNF, AKT1, CASP3, NOS3, and JUN through the AGE-RAGE, TNF, IL-17, and Toll-like receptor signaling pathways. PPAR*γ* seems to be a protective target gene during the process of pSS. These findings provide further evidence towards revealing the potential mechanism of WP in the treatment of pSS. Furthermore, they provide a reference for the development of new drugs directly and describe the pathological mechanism of pSS indirectly.

## Figures and Tables

**Figure 1:** A flow diagram predicting the potential mechanisms of WP against pSS.

**Figure 2:** The 32 overlapping target genes represent the potential therapeutic targets of WP against pSS. (a) A Venn diagram of intersecting target genes. (b) The PPI network graphic containing 32 nodes and 185 edges.

**Figure 3:** The D-D-I-T network map. Red hexagon represents WP, green circle represents SS, pink diamonds represent the active ingredients of WP, and the small blue ovals represent 32 overlapping target genes.

**Figure 4:** Further topological analysis of 32 overlapping target genes. Seven core targets were screened out and are listed in the center of the image.

**Figure 5:** (a) The top 20 enriched GO analysis items of core targets. (b) The top 20 enriched KEGG analysis signaling pathways of core targets.

**Figure 6:** The AGE-RAGE signaling pathway of core targets. Red represents the targets of the action of WP in the network.

**Figure 7:** The docking models of paeoniflorin binding to core targets. (a) IL-6, (b) TNF, (c) PPAR*γ*, (d) AKT1, (e) CASP3, (f) NOS3, and (g) JUN.

**Table 1:** Active ingredients of WP.

No.	Molecule ID	Molecule name	Molecular weight	OB (%)	DL
1	MOL001910	11alpha, 12alpha-epoxy-3beta-23-dihydroxy-30-norolean-20-en-28, 12beta-olide	470.71	64.77	0.38
2	MOL001918	Paeoniflorgenone	318.35	87.59	0.37
3	MOL001919	DPHCD	358.52	43.56	0.53
4	MOL001921	Lactiflorin	462.49	49.12	0.8
5	MOL001924	Paeoniflorin	480.51	53.87	0.79
6	MOL001925	paeoniflorin_qt	318.35	68.18	0.4
7	MOL001928	albiflorin_qt	318.35	66.64	0.33
8	MOL001930	Benzoyl paeoniflorin	584.62	31.27	0.75
9	MOL000211	Mairin	456.78	55.38	0.78
10	MOL000358	Beta-sitosterol	414.79	36.91	0.75
11	MOL000359	Sitosterol	414.79	36.91	0.75
12	MOL000422	Kaempferol	286.25	41.88	0.24
13	MOL000492	(+)-catechin	290.29	54.83	0.24

OB: oral bioavailability; DL: drug-likeness; DPHCD: (3S, 5R, 8R, 9R, 10S, 14S)-3, 17 dihydroxy-4, 4, 8, 10, 14-pentamethyl-2, 3, 5, 6, 7, 9-hexahydro-1HCyclopenta(a)phenanthrene-15, 16-dione.

**Table 2:** Seven core target genes of WP against pSS.

No.	Target	Entrez ID	BC	CC	DC
1	IL-6	3569	200.485	0.886	27
2	TNF	7124	109.839	0.816	24
3	PPAR*γ*	5468	81.383	0.795	23
4	AKT1	207	70.632	0.775	22
5	CASP3	836	29.046	0.721	19
6	NOS3	4846	36.928	0.705	18
7	JUN	3725	33.698	0.705	18

BC: betweenness centrality; CC: closeness centrality; DC: degree centrality.

**Table 3:** Docking energies.

Target	Paeoniflorin (kcal/mol)	Kaempferol (kcal/mol)	Beta-sitosterol (kcal/mol)
IL-6	−7.1	−6.7	−6.6
TNF	−9.1	−7.9	−7.8
PPAR*γ*	−9.2	−8.2	−7.6
AKT1	−8.8	−8.5	−7.6
CASP3	−7.8	−7.7	−9.9
NOS3	−9.7	−10.0	−8.6
JUN	−8.4	−9.2	−7.0

## Data Availability

The data used to support the findings of this study are available from the corresponding author upon request.
